This article has been retracted.

# Establishment of a Nomogram for Predicting Early Death in Viral Myocarditis

**DOI:** 10.1155/2021/9947034

**Published:** 2021-05-12

**Authors:** Xuejun Sun, Naxin Xie, Mengling Guo, Xuelian Qiu, Hongwei Chen, Haibo Liu, Hongmu Li

**Affiliations:** ^1^Department of Cardiovascular Surgery, Fujian Medical University Affiliated First Quanzhou Hospital, Quanzhou, China; ^2^Department of Medical Record, Fujian Medical University Affiliated First Quanzhou Hospital, Quanzhou, China; ^3^Department of Pharmacy, Fujian Medical University Affiliated First Quanzhou Hospital, Quanzhou, China

## Abstract

**Objective:**

This research aimed to establish a nomogram for predicting early death in viral myocarditis (VMC) patients.

**Method:**

A total of 362 consecutive VMC patients in Fujian Medical University Affiliated First Quanzhou Hospital between January 1, 2009, and December 31, 2019, were included. A least absolute shrinkage and selection operator (LASSO) regression model was used to detect the risk factors that most consistently and correctly predicted early death in VMC. The performance of the nomogram was assessed by calibration, discrimination, and clinical utility.

**Result:**

9 factors were screened by LASSO regression analysis for predicting the early death of VMC. Combined with the actual clinical situation, the heart failure (HF) (OR: 2.13, 95% CI: 2.76–5.95), electrocardiogram (ECG) (OR: 6.11, 95% CI: 1.05–8.66), pneumonia (OR: 3.62, 95% CI: 1.43–9.85), brain natriuretic peptide (BNP) (OR: 4.66, 95% CI: 3.07–24.06), and lactate dehydrogenase (LDH) (OR: 1.90, 95% CI: 0.19–9.39) were finally used to construct the nomogram. The nomogram's C-index was 0.908 in the training cohort and 0.924 in the validation cohort. And the area under the receiver operating characteristic curve of the nomogram was 0.91 in the training cohort and 0.924 in the validating cohort. Decision curve analysis (DCA) also showed that the nomogram was clinically useful.

**Conclusion:**

This nomogram achieved an good prediction of the risk of early death in VMC patients.

## 1. Introduction

Viral myocarditis (VMC) is one of the common clinical cardiovascular diseases, which is caused by viral infection, especially the localized or diffuse myocardial inflammatory lesions caused by Coxsackie B virus [1]. The potential pathogenesis was considered to be that the virus-mediated immune response can directly act on cardiomyocytes and intracardiac capillaries, leading to degeneration and necrosis of cardiomyocytes and ultimately injury cardiac dysfunction [2, 3]. The prognosis of most cases is good, but a small number of patients can have an acute outbreak leading to heart failure or sudden death, a small number of patients keep the heart cavity enlarged for several months to several years without heart failure, or the condition deteriorates again and evolves into dilated myocarditis [4, 5].

At present, there is no uniform standard for the diagnosis of viral myocarditis. Due to the lack of specificity in the clinical manifestations of viral myocarditis and most auxiliary examinations, the pathogenesis is not fully understood and the treatment is not satisfactory [6, 7]. There are no effective and safe preventive measures against early death from viral myocarditis. Therefore, accurate prognostic assessment will help doctors understand the early death risk of patients with viral myocarditis and take timely intervention measures to increase the survival probability of patients. However, there is no predictive model with good predictive ability for early death in VMC patients till now.

In this study, we retrospectively analyzed the existing case data to find the key factors for early death of viral myocarditis, build a nomogram to evaluate the severity of the patient's condition at the time of admission, and adopt corresponding treatment methods to reduce early death.

## 2. Patients and Methods

### 2.1. Patients

The study was approved by the Ethics Committee of Quanzhou First Hospital Affiliated to Fujian Medical University. A total of 362 consecutive hospitalizations of patients who were clinically diagnosed with VMC from January 1, 2009, to December 31, 2019, were included. The patients included in the study must be finally diagnosed with VMC, referring to the diagnostic guidelines of the Chinese Medical Association [8, 9], and the case data are complete. According to the clinical outcome at the time of discharge, they are divided into the survival group and death group (Figure 1).

### 2.2. Statistical Analysis

All statistical analysis was performed with R Studio software (Version 3.6.3, https://rstudio.com/). The least absolute shrinkage and selection operator (LASSO) regression method was used to detect the related risk factors in VMC [10, 11]. The “rms” package for *R* was used to make the nomogram. The accuracy of the nomogram was assessed by the discrimination ability and the calibration plot in the training set and the validating set [12]. AUC of receiver operating characteristic (ROC) was used to evaluate the discrimination ability of the nomogram. Decision curve analysis (DCA) was performed to evaluate the clinical utility of the nomogram [13, 14]. All tests were two-tailed, and *p* < 0.05 was considered statistically significant.

## 3. Result

### 3.1. Training Cohort's Characteristics

A total of 362 VMC patients visiting our clinic from January 1, 2009, to December 31, 2019, were assigned to training cohort. According to the principle of random allocation, 254 cases were screened for eligibility as the training cohort. Another 94 patients were enrolled into as validation cohort. There was no significant difference in demographic and clinical characteristics between the two groups, as given in Table 1.

### 3.2. Selection of Predictors for Early Death in VMC Patients

LASSO regression analyzed was performed to reduce 26 variables to 9 potential predictors in the training cohort (Figures 2(a) and 2(b)). However, only 5 predictors were enrolled into nomogram after combined with the actual clinical situation, including HF (OR: 2.13, 95% CI: 2.76–5.95), ECG (OR: 6.11, 95% CI: 1.05–8.66), pneumonia (OR: 3.62, 95% CI: 1.43–9.85), BNP (OR: 4.66, 95% CI: 3.07–24.06), and LDH (OR: 1.90, 95% CI: 0.19–9.39). The results of multivariate logistic analysis are presented in Table 2.

### 3.3. Nomogram Construction and Performance

A nomogram was constructed for predicting early death in VMC patients (Figure 3). Validation of the nomogram was performed with a 1000 bootstrap analysis. Harrell's concordance index was 0.908 in the training cohort and 0.924 in the validation cohort. The calibration curves of the nomogram showed good probability consistencies between the prediction and observation in the training cohort and validating cohort (Figures 4(a) and 4(b)). The area under ROC curve of the probability of early death was 0.91 in the training cohort and 0.92 in the validating cohort (Figures 4(c) and 4(d)).

### 3.4. Clinical Utility of the Nomogram

Decision curve analysis (DCA) was used to evaluate the clinical value of the nomogram using the data from all 362 patients. The DCA curve for the predictive nomogram is shown in Figure 5, which shows that when the nomogram-predicted probability of early death was <66%, the nomogram provided additional value relative to the treat-all-patients scheme or the treat-none scheme, suggesting that the nomogram was clinically useful.

## 4. Discussion

Viral myocarditis (VMC) is caused by various viruses infecting the myocardium, most of which have a good prognosis [3]. However, it has been linked as the cause of sudden cardiac death in young adults in up to 12% of cases [15, 16]. Little is known about the early stages of VMC in humans currently [7, 17]. There is no model with good predictive ability for early death in VMC patients till now.

In the present study, a nomogram was established to predict early death based on the clinical features of patients with VMC. 5 predictors were used to establish the nomogram, which included HF, ECG, pneumonia, BNP, and LDH. Finally, the nomogram provided good discrimination and calibration values, which may help to timely intervene in patients with VMC who are at high risk of early death.

HF is a consequence of various cardiovascular diseases, always associated with poor prognosis [18]. In this study, VMC patients with heart failure had a higher probability of early death. In addition, abnormal ECG is a strong prognostic indicator in the nomogram. However, Dec et al. suggested that ECG findings are neither sensitive nor specific for the diagnosis of myocarditis [19], which requires further exploration.

Zhang et al. [20] suggested that levels of brain natriuretic peptide (BNP) measured in the plasma could be a useful biochemical marker for the myocarditis, and high concentration of BNP may correlate with poor prognosis in patients with myocarditis. Thus, pneumonia and LDH elevated seemed to be an important sign of early death in VMC patients. However, no correlation with prognosis was found in previous studies.

In this study, the levels of CK, CK_MB, and TNI_I were not significant for early death. However, a significant increase in TNI_I may suggest a worse prognosis [21].

There are also several limitations of this research. First, this study was dependent on the data of a single institutional cohort of patients from the Asia-Pacific region. Second, this retrospective study was susceptible to certain biases that could not be completely avoided. Third, in medical practice, instead of applying endomyocardial biopsy (EMB), the current gold standard for diagnosis [22], physicians rely on a combination of clinical features, laboratory analyses, and imaging to diagnosis VMC.

## 5. Conclusion

In conclusion, we established and validated a nomogram for predicting early death in VMC patients. The nomogram has an adequate ability of discrimination, calibration, and may be a valuable tool for clinical practice.

## Figures and Tables

**Figure 1:** Research plan and implementation flow chart.

**Figure 2:** Lasso regression analysis was used to screen the potential predictors. (a) The results without cross-validation. (b) The results after cross-validation.

**Figure 3:** The nomogram for preoperative prediction of early death in viral myocarditis (VMC) patients.

**Figure 4:** The performance of the nomogram. Calibration plot of the nomogram in (a) the training cohort and (b) validation cohort. The receiver operating characteristic (ROC) curves of the nomogram in (c) the training cohort and (d) the validation cohort.

**Figure 5:** Decision curve analysis for the nomogram.

**Table 1:** Demographic and clinical characteristics of all patients.

Variables	Training cohort (*n* = 254)		Validation cohort (*n* = 108)		*P* value
	Early death (25)	Survival (229)	Early death (10)	Survival (98)	
Age (>60 y)	16 (64.00)	154 (67.25)	8 (80.00)	67 (68.37)	>0.05
Male	15 (60.00)	143 (62.44)	4 (40.00)	60 (61.22)	>0.05
Smoking	5 (20.00)	34 (14.85)	0 (0.00)	21 (21.43)	<0.05
Drinking	17 (68.00)	175 (76.42)	8 (80.00)	67 (68.37)	>0.05
Hypertension	1 (4.00)	16 (9.99)	1 (10.00)	5 (5.10)	>0.05
Diabetes	0 (0.00)	5 (2.18)	1 (10.00)	2 (2.04)	>0.05
HF	9 (37.04)	25 (10.92)	4 (40.00)	8 (8.16)	>0.05
Abnormal ECG	10 (40.00)	180 (78.60)	10 (100.00)	17 (17.35)	<0.05
Pneumonia	17 (68.00)	55 (24.02)	8 (80.00)	25 (25.51)	>0.05
WBC (>9.5 × 10^∧^9/L)	16 (64.00)	103 (44.98)	10 (100.00)	49 (50.00)	>0.05
*N*% (>75%)	20 (80.00)	100 (43.67)	8 (80.00)	48 (48.98)	>0.05
Lymphocyte >3.2 × 10^∧^9/L	7 (28.00)	9 (3.93)	2 (20.00)	6 (6.12)	>0.05
Monocyte >0.6 × 10^∧^9/L	11 (44.00)	51 (22.27)	3 (30.00)	28 (28.57)	>0.05
Hb < 120 g/L	6 (24.00)	30 (13.10)	0 (0.00)	12 (12.24)	>0.05
PLT <100 × 10^∧^9/L	8 (32.00)	29 (12.66)	5 (50.00)	24 (24.49)	>0.05
BNP ≥500 pg/L	24 (96.00)	80 (34.93)	9 (90.00)	36 (36.73)	>0.05
TNI_I > 0.5 ng/ml	23 (92.00)	140 (61.14)	8 (80.00)	65 (66.33)	>0.05
TP < 65 g/L	6 (24.00)	10 (4.37)	2 (20.00)	3 (3.06)	>0.05
Albumin<40 g/L	4 (16.00)	28 (12.23)	3 (30.00)	8 (8.16)	>0.05
ALT >50 U/L	19 (76.00)	101 (44.10)	7 (70.00)	42 (42.86)	>0.05
AST >40 U/L	22 (88.00)	110 (48.03)	7 (70.00)	50 (51.02)	>0.05
LDH ≥300 U/L	24 (96.00)	110 (48.03)	8 (80.00)	55 (56.12)	>0.05
CK > 200 U/L	25 (100.00)	193 (85.77)	8 (80.00)	87 (88.78)	>0.05
CK_MB > 25 U/L	23 (92.00)	146 (63.76)	7 (70.00)	70 (71.43)	>0.05
Cr ≥110 umol/L	11 (44.00)	28 (12.22)	6 (60.00)	10 (10.20)	>0.05
UA >500 umol/L	10 (40.00)	67 (29.26)	6 (60.00)	20 (20.41)	>0.05

HF, heart failure; ECG, electrocardiogram; WBC, white blood cell count; *N*%, neutrophil percentage; Hb, hemoglobin; PLT, platelet; BNP, brain natriuretic peptide; TP, total protein; TNI_I, Troponin I; ALT, alanine aminotransferase; AST, aspartate aminotransferase; LDH, lactate dehydrogenase; CK, creatine kinase; CK-MB, creatine kinase, MB form; Cr, creatinine; UA, uric acid.

**Table 2:** Prediction factors for early death in VMC patients.

Intercept and variable	Prediction model		
	*β*	Odds ratio (95% CI)	*P* value
Intercept	−8.52	0.04 (95% CI:0.00–0.16)	*P* < 0.05
HF	0.45	1.57 (95% CI:1.86–4.73)	*P* > 0.05
ECG (abnormal)	2.14	8.49 (95% CI:1.42–12.34)	*P* > 0.05
Pneumonia	1.14	3.11 (95% CI:1.14–9.02)	*P* < 0.05
BNP (≥ 500 pg/L)	2.68	3.97 (95% CI:2.70–20.10)	*P* < 0.05
LDH (≥ 300 U/L)	0.63	1.87 (95% CI:2.45–5.22)	*P* > 0.05

HF, heart failure; ECG, electrocardiogram; BNP, brain natriuretic peptide; LDH, lactate dehydrogenase.

## Data Availability

The data used to support the findings of this study are included within the article and within the supplementary files.

## Supplementary Materials

Supplementary Materials Supplementary Table 1. Original data of training cohort. Supplementary Table 2. Original data of validation cohort. Supplementary Table 3. Original script.
